This article has been retracted.

# Provisional Decision-Making for Perioperative Blood Pressure Management: A Narrative Review

**DOI:** 10.1155/2022/5916040

**Published:** 2022-07-11

**Authors:** Qiliang Song, Jipeng Li, Zongming Jiang

**Affiliations:** Department of Anesthesiology, Shaoxing People's Hospital (Shaoxing Hospital, Zhejiang University School of Medicine), Shaoxing, 312000 Zhejiang Province, China

## Abstract

Blood pressure (BP) is a basic determinant for organ blood flow supply. Insufficient blood supply will cause tissue hypoxia, provoke cellular oxidative stress, and to some extent lead to organ injury. Perioperative BP is labile and dynamic, and intraoperative hypotension is common. It is unclear whether there is a causal relationship between intraoperative hypotension and organ injury. However, hypotension surely compromises perfusion and causes harm to some extent. Because the harm threshold remains unknown, various guidelines for intraoperative BP management have been proposed. With the pending definitions from robust randomized trials, it is reasonable to consider observational analyses suggesting that mean arterial pressures below 65 mmHg sustained for more than 15 minutes are associated with myocardial and renal injury. Advances in machine learning and artificial intelligence may facilitate the management of hemodynamics globally, including fluid administration, rather than BP alone. The previous mounting studies concentrated on associations between BP targets and adverse complications, whereas few studies were concerned about how to treat and multiple factors for decision-making. Hence, in this narrative review, we discussed the way of BP measurement and current knowledge about baseline BP extracting for surgical patients, highlighted the decision-making process for BP management with a view to providing pragmatic guidance for BP treatment in the clinical settings, and evaluated the merits of an automated blood control system in predicting hypotension.

## 1. Introduction

Approximately 300 million surgical operations are conducted globally every year [1, 2], with most of the concerned patients being at risk of perioperative hemodynamic instability. The American College of Cardiology/American Heart Association (ACC/AHA) updated its guidelines for blood pressure (BP) management in patients with chronic hypertension in 2017, and the European Society of Cardiology/European Society of Hypertension updated its guidelines in 2018 [3, 4]. However, these guidelines are not fully applicable to perioperative patients because of the dynamic nature of the patients' physiological status, characterized by increased stress and immune response, inflammation, hypercoagulable state, and pain [5–8]. For long, anesthesiologists have been taught and believed that perioperative BP should be maintained within ±20% of the baseline values in practice; however, this recommendation is not evidence-based. Consequently, BP management varies considerably among clinicians. To provide pragmatic guidance and highlight the importance of optimizing BP perioperatively, this manuscript is a review of recent research on perioperative BP management, especially those on the targets and decision-making process.

## 2. The Physiology of BP and Organ Perfusion

BP is one of the routinely measured variables in the perioperative period; it is the force that propels blood to the tissues and organs. BP is the interplay between cardiac output or stroke volume and systemic vascular resistance at a given filling pressure, which is affected by various hemodynamic elements [5] such as intravascular volume, myocardial contractility, cardiac compliance, heart rate, and vascular radius (Figure 1). A change in one or more of these elements will not necessarily cause a change in BP. Besides, biological rhythms, hormones, and emotional states can also affect BP [9, 10]. BP is an important determinant for organ blood flow supply. Insufficient blood supply causes tissue hypoxia, provokes cellular oxidative stress, and leads to organ injury and even dysfunction to some extent. The BP levels that trigger cellular oxidative stress or tissue injury vary with organs. Therefore, the underlying pathophysiological mechanisms of hypotension or hypertension may be individualized and have different influences on organ perfusion.

Pressure autoregulation is a self-regulation mechanism of an organ to maintain stable perfusion amidst fluctuations in BP or perfusion pressure [11]. When BP fluctuates violently and exceeds the pressure autoregulation threshold, the organs get into a hypo/hyperperfusable state. Of course, the autoregulation ability varies with organs, a feature known as heterogeneity. Vital organs (the brain, heart, kidneys, and spinal cord) have robust pressure autoregulation mechanisms. In contrast, the visceral organs, such as the stomach, small intestines, and colon, have weaker pressure autoregulation mechanisms, which bear the brunt when BP fluctuates violently [12]. Besides, pressure autoregulation is also influenced by intraindividual heterogeneity factors including age, chronic or acute disease, anesthesia, and sympathetic tone [12]. For example, the lower threshold of cerebral perfusion pressure in healthy participants varies from a mean arterial pressure (MAP) of 53 to 113 mmHg, with a gap of up to 60 mmHg [13].

Organ perfusion is regulated by perfusion pressure and organ-specific resistance. Perfusion pressure is determined by the gradient between the upstream pressure and downstream pressure (Figure 1). MAP decreases progressively from central to peripheral arteries given the relatively low resistance of the arterial system. Hence, MAP is a reference for organ input pressure [5]. Organ perfusion depends on BP via pressure autoregulation and the cardiac output among organs, since the total perfusion shared by all organs is equal to the cardiac output [14]. Decreased cardiac output results in blood flow redistribution to different organs, with vital organs being prioritized [15]. In a previous study, this kind of blood flow redistribution was examined in cardiac surgery; it was observed that compared to a low MAP (40–50 mmHg), a higher MAP (70–80 mmHg) did not significantly decrease the severity of brain infarcts diagnosed postoperatively [16]. This is explained by the fact that the same laminal pump flow of 2.4 L min^−1^2009m^−2^, which provides the same cardiac output, was used for both groups. Even though the BP was much lower in the low MAP group, the perfusion of the brain was well guaranteed. In contrast, the BP was maintained within the normal range in the perioperative period by surgical stress or vasopressor infusion, which may mask insufficient organ perfusion due to decreased cardiac output. Therefore, the goal of perioperative BP management is to optimize adequate blood flow supply, not just to concentrate on the BP values.

## 3. Perioperative BP Monitoring and Baseline BP

Appropriate BP monitoring is a prerequisite for obtaining accurate BP values and providing reliable guidance for perioperative BP management. The two most used methods for BP monitoring are intermittent oscillometric manometry with a noninvasive cuff and continuous intra-arterial invasive catheterization; however, cuffless BP measurement is an emergent popular field due to the clinical need and technology advances [17, 18]. Intraoperative BP is measured using intermittent oscillometric manometry [19], which allows automatic, intermittent BP measurement, usually at 3–5 min intervals. The measurement accuracy depends on the selection of a suitable cuff that matches the circumference of the patients' biceps, patients' posture and ambient temperature, etc.

Continuous intra-arterial invasive manometry is performed using intraperipheral arterial cannula placement, which allows for continuous, real-time, and accurate BP measurement. Conventionally, it is believed that the accuracy of BP measured invasively is more than that measured with cuffs, and invasive BP measurements are often regarded as the reference method due to cuff pressure shows large limits of agreement compared to invasive BP [20]. However, there may be differences between noninvasive cuff pressure and invasive arterial pressure in different situations. In a study by Wax et al. [21] involving 24225 patients, the BP of 63% of the patients were measured both noninvasively (cuff BP) and invasively (radial artery BP), while that of 37% was measured only invasively (radial artery BP). They observed that in patients with hypotension, particularly those with an arterial systolic BP below 111 mmHg, the noninvasive cuff BP was higher than the invasive arterial pressure in most cases. However, in the patients with hypertension, the invasive measurements were higher than the noninvasive cuff pressure in most cases, especially the systolic BP values [22]. This is mainly because of the amplification of the pulse pressure difference as the pulse wave propagates from the aorta to the peripheral arteries [23], especially in patients with chronic hypertension. In patients receiving vasopressors, such as patients with sepsis [24], liver transplantation [25], and cardiac surgery under extracorporeal circulation [26], BP measured by invasive manometry is often lower than the central BP. In clinical settings, the noninvasive cuff pressure should be measured simultaneously when there is a significant difference between the two values, especially when the invasive BP is significantly low. Because the noninvasive cuff pressure is closer to the actual BP, it should be the basis for relevant management measures [27]. When encountering this condition, the merits of invasive BP should not be ignored and should be considered supplement for BP treatment.

In addition to accurate BP monitoring, obtaining a reliable and true baseline BP might be critical for BP titration and decision-making. As for the definition of baseline BP, it lacks standard definition and also varies with studies. Several studies [28–31] on the relationship between intraoperative hypotension (IOH) and BP-related complications reported that the BP value obtained before anesthesia induction should be considered the baseline BP; however, this definition is debatable and vague. Saugel et al. [9] selected patients under general anesthesia aged 40–65 years undergoing elective noncardiac surgery as the study population; they compared preoperative 24 h ambulatory BP with preanesthesia induction, postanesthesia induction BP, and intraoperative MAP. They observed that the correlation between the first BP value obtained before anesthesia induction and preoperative ambulatory MAP was poor (*r* = 0.429), which suggested that BP before anesthesia induction cannot be regarded as the baseline BP. To obtain an accurate baseline BP, Ard et al. [32] conducted a prospective and observational trial involving 2087 patients and measured the BP in three locations (surgical visiting clinic, unit for preoperative punctuality, and the first BP at the operating theatre). They observed that the BP obtained in the theatre was markedly higher (*P* < 0.01 for all comparisons), specifically systolic BP (138 ± 23 mmHg), diastolic BP (77 ± 14 mmHg), and MAP (97 ± 14 mmHg), whereas no difference was observed between the first two measurements with 128 ± 17 mmHg and 74 ± 11 mmHg and 124 ± 18 mmHg, 73 ± 11 mmHg, and 92 ± 12 mmHg, respectively. Consequently, they concluded that the BP before anesthesia induction could not be used as the baseline BP, while the BP measured in the preoperative holding area could be used as the baseline BP. Hu et al. had consistent findings with theirs [33]: the BP measured at the holding area before surgery was considered the baseline BP, and there was an association between baseline MAP and acute kidney injury (AKI) in patients after cardiac surgery, implying that this baseline BP could be used as an important predicting factor for AKI. To ascertain whether baseline BP obtained at different time points can optimize intraoperative brain function, Drummond et al. [34] defined the baseline BP as the average of three or more ambulatory clinic BP values 7 months earlier and compared them to the first BP measured in the operating cabinet in a retrospective study. They observed that if the first BP measured in the operating theatre was suggestive of hypertension, the BP was greater than ambulatory clinic recordings 7 months earlier. Furthermore, if the first BP was consistent with normotension, the BP reflected the baseline BP. Based on the previous literatures, a widely accepted protocol to determine awake baseline BP is to take BP measurement 3 to 5 times in the ward or visiting clinic after resting 5 to 10 minutes in a quiet and comfortable site, and the average of all readings can be regarded as baseline BP [35, 36].

Currently, it is hypothesized that the preoperative 24 h ambulatory BP is the best reflection of the daily BP, which can be used as the baseline BP [5]. However, performing 24 h ambulatory BP monitoring preoperatively for each surgical patient to obtain the baseline BP is not practical. Therefore, further research is needed to determine a clinically practical and easy method for determining baseline BP.

## 4. The Importance of Preoperative BP Optimization

Preoperative hypertension increases the risk of perioperative adverse events. The ACC/AHA guidelines recommend postponing any elective surgery for a patient with a preoperative BP above 180/110 mmHg [3, 4]. However, a previous study [37] revealed that there is no relationship between BP > 180/110 mmHg and perioperative adverse events. Moreover, there is no clear evidence that the delay in performing the surgery will improve perioperative outcomes. This is because for a timely surgery the BP should be titrated to the ideal level within a short preoperative time if it was delayed. Moreover, the rapid control of BP with medications increases the risk of postoperative complications, especially in patients with significantly elevated preoperative BP [38]. Consequently, Howell et al. [37] reported that surgery should not be delayed because of isolated elevated preoperative BP values only in a healthy patient. Certainly, a goal of ±20% baseline BP during surgery should be kept, and measures should be taken to ensure a stable cardiovascular system intraoperatively. On the other hand, the importance of preoperative BP optimization in patients with hypertension should not be ignored.

Commonly used antihypertensive agents include angiotensin-converting enzyme inhibitors, angiotensin receptor inhibitors, *β*-blockers, and calcium channel blockers. Studies have observed that angiotensin-converting enzyme inhibitors and angiotensin receptor inhibitors often complicate protracted IOH [39] and may increase the incidence of perioperative AKI, stroke, myocardial injury, and mortality [40]. Therefore, the Canadian Cardiovascular Society, the European Cardiovascular Society, and the European Society of Anesthesiologists recommend the discontinuation of both drugs on the day of surgery [4, 41, 42]. Patients with chronic *β*-blocker intake, especially those with congestive heart failure or recent myocardial infarction, can continue during the perioperative period [43, 44]. However, *β*-blockers may be deleterious in the perioperative period, as their intake is characterized by frequent hypotension and end-organ hypoperfusion. The 2008 PeriOperative ISchemic Evaluation (POISE) trial found that although preoperative initiation of *β*-blockers reduced the risk of nonfatal myocardial infarction, it increased the risk of cardiovascular adverse events (including bradycardia, stroke, and hypotension) and mortality in the perioperative period [45]. This finding was consistent with the results of a large retrospective cohort study, which showed that continuing *β*-blockers increased the 30-day mortality after surgery in elderly patients with hypertension having elevated systolic BP [46]. While Kertai et al. [47] found that although withdrawal of *β*-blockers reduced the need of vasopressor and shortened stay in the postanesthesia care unit, it increased risk for mortality within 48 hours after noncardiac surgery. Over the past 30 years, multiple studies have concerned about the best strategy for the perioperative approach to patients receiving *β*-blockers. Due to the use of *β*-blockers are not limited perioperatively, whether withholding or continuing and timing is still a debate and needs further study [48].

Preoperative hypotension also increases the risk of postoperative adverse events. Venkatesan et al. [7] found that preoperative systolic BP < 119 mmHg and diastolic BP < 63 mmHg were associated with increased 30-day mortality in elderly patients undergoing elective noncardiac surgery, lower preoperative BP, and higher postoperative mortality. Preoperative hypotension increases the incidence of IOH, decreases coronary perfusion pressure, and shifts the autoregulation curve to the left, which leads to ischemia of vital organs. Preoperative hypertension or hypotension in patients awaiting surgery should be normalized preoperatively, and aggressive BP management is needed to reduce or avoid adverse events.

## 5. Intraoperative BP Control Target and Its Implications

Hypotension is common during the operative period. However, the definition of IOH remains controversial. Bijker et al. [49] identified 140 definitions of IOH after a review of 130 articles. The most used definition of IOH was as follows: a decrease in the systolic BP of more than 20% from the baseline BP or a MAP < 65 mmHg [50, 51]. The latter, also known as absolute thresholds, is used more frequently for the following reasons: (1) baseline BP measurements are often unknown, and approximately one-third of patients do not have a baseline BP value preoperatively, as described by Monk et al. [28]; (2) relative thresholds are not superior to absolute thresholds in predicting unfavorable outcomes as reported by Salmasi et al. [52] in a large-sample retrospective cohort analysis; (3) absolute thresholds are concrete and easier to use in decision-making; and (4) preoperative BP measurements are often elevated due to tension and anxiety. Therefore, in daily practice, absolute thresholds are adopted frequently as the baseline for BP regulation.

IOH may lead to inadequate blood supply and various degrees of organ dysfunction. Several studies [16, 28, 52–76] found that IOH was associated with postoperative detrimental outcomes (such as AKI, myocardial injury, and neurocognitive disorders), which is related to the duration and magnitude of hypotension [77], suggesting that IOH should be avoided perioperatively (Table 1). Based on existing evidence [51, 56, 58, 74, 75], intraoperative MAP should be maintained above 65 mmHg in normal adult patients, and in patients with other comorbidities (for example, coronary artery disease and carotid stenosis), the intraoperative MAP must be individualized based on the patient's pathophysiology and clinical situation. For example, the MAP of patients with chronic hypertension should be maintained above 70 mmHg. Of note, the advocation of absolute thresholds in BP management does not mean that one-size-fits-all methods should be used. Conversely, it will lead to hypoperfusion. For instance, in chronic hypertension cases, the autoregulatory mechanisms of the kidneys are likely compromised [78], with a right shift of the threshold [79, 80]. Therefore, higher MAP values should be maintained to ensure sufficient blood flow. A combination of absolute thresholds in BP management and individualized BP tailoring should be implemented for patients with comorbidities.

## 6. Postoperative BP Management

Postoperative BP is a basic component of the perioperative period, and its appropriate management is essential for a smooth postoperative recovery. Postoperative hypotension (POH) management is an important component of postoperative BP management [81].

Considering the controversy in POH, the incidence of POH varies considerably (from 8%–48%) when based on different MAP thresholds of 60–75 mmHg [82]. The secondary analysis from the POISE-2 trial [54] showed that the incidence of POH was 7.6% in the first four postoperative days. There are very few studies on the association between postoperative BP and organ insufficiency. Recent studies have shown that POH contributes to the occurrence of myocardial injury [40, 82, 83] and infarction [54]. To the best of our knowledge, the optimal postoperative BP target and BP threshold that leads to organ injury remains unclear [84]. Besides, duration of POH > 10 min is associated with increased risk of postoperative myocardial infarction and 30-day mortality in elderly patients. Furthermore, longer duration and greater magnitude of hypotension (systolic BP < 90 mmHg) significantly increase the risk of myocardial injury [54]. Similarly, Mohammed et al. [85] and Kause et al. [86] also observed that systolic BP < 90 mmHg was associated with postoperative emergency events in the general ward. Based on existing literature [82, 87, 88], POH is an independent surrogate predictor for postoperative myocardial injury, and avoiding POH helps to attenuate myocardial injury.

Whether there are causal interactions between POH and IOH is unclear. To ascertain the severity of IOH on the occurrence of POH and outcomes, a study involving 2833 patients who were transferred to the surgical intensive care unit postoperatively was conducted to investigate whether there is an association between hypotension and cardiovascular incidents or death within seven postoperative days; there was a strong association between POH and IOH severity, especially the lowest intraoperative MAP [89]. Contrarily, a retrospective study conducted in 2008–2017 and involving 67968 patients (with POH and not IOH) undergoing noncardiac surgery was conducted to assess the relationship between major adverse cardiovascular or cerebrovascular events within 30 postoperative days [90]; it was revealed that in the patients without IOH, POH was not associated with major adverse cardiovascular or cerebrovascular events at any MAP threshold (≤75, ≤65, and ≤55 mmHg). Therefore, they suggested that there was no interaction between POH and IOH. Notably, due to the inherent study limitations and the few patients with a MAP below 55 mmHg, the applicability of the conclusion in clinical practice is limited. Further studies are necessary to assess the interactions between POH and IOH.

Timely detection and prompt intervention is essential in POH correction. In the general ward, unlike the conditions in the operating theatre, monitoring of vital signs is usually intermittent with 30 min to 4–6 h intervals. Therefore, POH is often ignored or undetected during the monitoring; approximately 50% of the patients with POH are not identified, and if they are identified, it implies that the POH has been ongoing for a long time [91]. Given this situation, there is a growing interest in continuous monitoring of patients postoperatively in the general ward, which allows earlier detection of POH and thus prompt treatment, improved patient outcomes, and fewer resuscitation events, especially for high-risk patients [92–94]. Besides, stopping antihypertensive medication preoperatively favors postoperative BP management. When and how to initiate antihypertension agents should be weighted based on risks and benefits [41, 42, 84].

## 7. Individualized Hemodynamic Management in Perioperative Care Is Promising

In the past decades, BP thresholds from popular studies were used as therapeutic targets for perioperative BP management. A BP management strategy using one-size-fits-all principles does not represent an accurate personalized BP threshold for organ perfusion and oxygen supply. The current ACC/AHA guidelines [44] recommend individualized care for noncardiac surgical patients with associated comorbidities.

With the rapid advances in medical science and improved disease knowledge, perioperative individualized BP management is attracting clinical attention [73, 95–97]. Perioperative individualized BP management could be defined as intraoperative BP target values based on each patient's physiological and surgical characteristics, while considering acute and chronic pathophysiological cardiovascular alterations [98].

In 2017, a randomized clinical trial involving 678 elderly patients with hypertension who underwent major gastrointestinal operations were enrolled into three MAP groups (65–79, 80–95, and 96–110 mmHg) receiving intraoperative goal-directed fluid therapy (stroke volume variation: 8%–13%). Also, four vasopressor agents were used to titrate BPs within the target range. This suggested that a MAP level of 80–95 mmHg markedly lowers the possibility of postoperative AKI [69]. Intriguingly, an intermediate MAP is conducive for postoperative renal function recovery, although the authors assigned the patients to three preset MAP groups arbitrarily, suggesting that strict BP control is beneficial for organ functioning in patients with a normal BP range. Similarly, in a multicenter randomized study, 322 elderly patients were assigned to two groups based on intraoperative MAP levels (60–70 or 90–100 mmHg), and the results concluded that a high MAP significantly reduces the occurrence of postoperative delirium [66]. In nonsurgical patients, the BP management strategy affects cognitive function, and a good control for hypertension reduces the risk of cognitive impairment. In this regard, patients with Alzheimer's disease were randomly allocated into standard BP control (systolic BP goal < 120 mmHg) or intensive BP control (systolic BP goal < 140 mmHg) groups; the latter was associated with a mild and significant decrease in cerebral volume [99]. This might be the robust evidence supporting the fact that BP control and intensive BP may influence cerebral volume better than standard care in patients with hypertension.

Individualized BP control considering baseline BP might meet the demands for individuals, and perioperative BP should be tailored in an individual pattern. Futier et al. [73] pioneered individualized BP tailoring in 2017, and in their study, the eligible patients were randomly allocated into individualized BP management groups (systolic BP was controlled within 10% of the baseline value during surgery under the administration of norepinephrine) and conventional BP management group (ephedrine was injected when the systolic BP was less than 80 mmHg or was 40% lower than the preoperative values). They observed that individualized BP management reduced the incidence of systemic inflammatory response syndrome; renal, cardiovascular, coagulation, or neurological impairment; or impairment of at least one vital organ system, compared to routine management [73]. However, this study did not evaluate the volume status objectively. Titration of vasoconstrictors to maintain individualized arterial pressure might cover the hypovolemic status, which would reduce end-organ blood flow and result in tissue hypoperfusion.

Lately, individualized hemodynamic management requiring optimizing the volume simultaneously during individualized BP management was introduced into clinical practice [100]. Typically, this entails using a closed-loop autonomous system and incorporating machine learning (a subset of artificial intelligence) to control and predict BP variations during the operative period. In a randomized clinical trial on individualized hemodynamic management published in 2020, 188 high-risk patients undergoing major abdominal surgery were divided into a conventional management group and an individualized management group, which required anesthesiologists to use a proprietary algorithm, based on a noninvasive pulse wave analysis to guided intraoperative fluid infusion and/or dobutamine administration, thus maintaining the intraoperative cardiac index at the baseline values. The results showed that the individualized management group had a lower composite outcome of major postoperative complications or death within 30 days [97]. In 2021, Joosten et al. [101] developed a hybrid system including a computer-assisted closed-loop system for vasopressors and a decision-support system for bolus fluid challenge for intermediate to high-risk surgical patients. They observed that the prevalence of IOH in the computer-assisted group was 1.2% and 21.5% in the individualized management group. This suggests that individualized hemodynamic optimization decreases the incidence of IOH and may be a potential BP management strategy.

Fundamentally, there are frequent serial fluctuations in cardiocirculatory parameters prior to hypotension. Hence, the development of a hypotension prediction index will help prevent hypotension. By analyzing BP waveform characteristics using machine deep learning algorithms, Hatib et al. [102] pioneered the prediction of hypotension occurrence with MAP values below 65 mmHg 1 min, 5 min, or even earlier, thus allowing clinicians to intervene during hypotension or even prevent hypotension. The algorithm was verified in 204 surgical patients. It showed that the sensitivity and specificity of predicting hypotension 15 min before the onset of hypotension were 88% and 87%, respectively. However, the algorithm was unable to predict hypotension due to clinical interventions, including intraoperative compression of large vessels or changes in position, such as the Trendelenburg position. Schneck et al. [103] found that the application of the algorithm conferred a significantly lower IOH incidence and a significantly shorter IOH duration than conventional BP management. However, in a single-center trial by Maheshwari et al. [104] involving 214 patients undergoing medium- and high-risk noncardiac surgery, the algorithm predicted hypotension but did not reduce the amount of IOH. The investigators concluded that the algorithm for treatment recommendations in the treatment algorithm system was too complex and needed further optimization to ensure timely clinical intervention. Based on this, considering the large proportion of low-risk patients who undergo conventional common surgery, we should weigh the risk-benefit ratio when using expensive noninvasive hemodynamic devices, as it is a valuable tool or a superfluous toy for the right patients [105]. Fully automated individualized hemodynamic management has broad prospects with advances in computer technology, especially in high-risk patients, as supported by recent studies [75, 106, 107].

## 8. Provisional Decision-Making and Targets in Practice

Given the dynamic nature of BP, perioperative individualized BP management is not to set a fixed threshold, but rather an individualized BP target value that considers the baseline BP, pathophysiology, comorbidities, perioperative agent use, and surgery.

In clinical practice, individualized BP targets can be achieved, which will ultimately improve patient outcomes through an easy and rapid process. The “5 Ts” (target patients, timing and type of intervention, target variables, and values) may provide a reference for rapid individualized BP management [108, 109].

Targeting an appropriate BP is a challenge. Clinically, several factors should be considered when setting an appropriate BP target [110, 111]: (1) hypotension does not always appear to be harmful and lead to organ hypoperfusion [112]; (2) the goal is to ensure sufficient perfusion pressure and oxygen delivery, not to correct a number [113]; (3) the pressure regulation ability and ischemia tolerability varies with organs [110, 111]; (4) an absolute threshold is easy to use and often adopted in decision-making; (5) intravascular volume status is fundamental and essential for organ perfusion and should be evaluated simultaneously when correcting hypotension [114, 115]; (6) specific pathophysiology alterations of the surgical patient (e.g., shock, hemorrhage, and sepsis); (7) the BP requirements for high-risk elderly patients undergoing major surgery is quite different from those of normal patients undergoing a brief surgery; (8) strict BP management is more conducive for the protection of organ functions than laissez-faire or lenient BP management [116]; (9) a “one-size-fits-all” approach should be abandoned and personalized BP targets that vary with time should be adopted; and (10) a holistic attitude when treating refractory hypotension should be adopted.

BP targets vary with the population characteristics and surgical type. The patient's baseline BP measurements are a major determinant for perioperative BP targets. Based on the BP values, the baseline BP can be classified into three categories: the low (systolic BP < 90 mmHg and diastolic BP < 50 mmHg), normal (systolic BP 90–139 mmHg and diastolic BP 50–89 mmHg), and high baseline BP (systolic BP ≥ 140 mmHg and diastolic BP ≥ 90 mmHg) categories. The BP target for patients with a low baseline BP undergoing noncardiac surgery should be maintained at a MAP ≥ 60 mmHg based on results of multiple studies [52, 55–57, 64] and a MAP > 65 mmHg for patients with a normal BP [30, 50, 73, 117]. BP should be maintained within 80%–110% of the baseline BP in patients with a high baseline BP [30, 52, 73, 118, 119] and at a systolic BP of ≤160 mmHg [63, 120], which is favorable for the outcomes. For cardiac surgery, the requirements for BP during and before or after extracorporeal circulation are different. Before and after extracorporeal circulation, the target BP may be the optimal value for patients undergoing noncardiac surgery: the intraoperative systolic BP should not be higher than 140 mmHg [50, 121], and the MAP should be kept at 70–100 mmHg during cardiopulmonary bypass [70, 71, 122, 123]. BP targets for patients with specific pathophysiological alterations should be tailored in an individualized manner. In a perioperative setting, two conditions are often encountered: the BP targets and management of hypotension. The pragmatic decision-making flow chart is depicted in Figure 2.

For postoperative BP, maintaining a systolic BP of 90–160 mmHg is a reasonable target for patients with a normal baseline BP. However, for patients with an abnormal baseline BP, these targets should be adjusted according to the preoperative baseline values [84].

## 9. Conclusion and Perspectives

BP can be corrected, and hypotension should be avoided. Given the nature of BP, perioperative BP management is a dynamic process and not a fixed point. From existing evidence, maintaining the MAP of normal patients at ≥65 mmHg perioperatively is widely accepted, MAP value at 65 mmHg can be considered a minimum level for BP management and adjustment and at the same time not solely concentrates on the value but tailors individually suffice for organ blood supply.

Both IOH and POH have detrimental effects on patient prognosis, and there is paucity of evidence on the direct relationship between hypotension and adverse outcomes, and an absolute BP target is usually selected as the initial target for perioperative BP management. The baseline BP is helpful for setting an appropriate BP target, and personalized BP targets may change over time owing to abrupt pathophysiological alterations perioperatively. Strict BP management relying on baseline BP and maintaining fluctuations within ±20% or ±10% of the baseline BP is an optimal BP control method. Further research is needed to define individual BP harm thresholds and to develop therapeutic strategies to treat and avoid IOH.

The newly emerged hypotension prediction index algorithm and automated BP control system are helpful for individualized hemodynamic management, especially for high-risk patients. It is necessary to validate whether the machine learning algorithm or artificial intelligence-based intervention for BP management is valuable for all patients, especially for high-risk patients.

## Figures and Tables

**Figure 1:** The physiology of BP and miscellaneous factors affecting organ perfusion. BP is determined by production of CO and SVR. PA: blood flow redistribution and organ-specific RVR influence the organ perfusion. BP: blood pressure; CO: cardiac output; SV: stroke volume; SVR: systemic vascular resistance; PA: pressure autoregulation; RVR: regional vascular resistance.

**Figure 2:** The flow chart for decision-making for BP targets and hypotension interventions during surgery. The main determinants for BP targets are baseline BP, type of surgery, and specific pathophysiological alterations and weight between organ ischemia and impending surgical bleeding. The BP targets are initial values and a fixed threshold, and maintaining sufficient oxygen supply is priority to a fixed BP value. Individualized BP management highlights the importance of balancing conflicting risks. BP: blood pressure; SBP: systolic blood pressure; DBP: diastolic blood pressure; MAP: mean arterial pressure; and CPB: cardiopulmonary bypass.

**Table 1:** Recent studies on the association between IOH and perioperative outcomes.

Author (year)	Study design	Study population	IOH definition	Baseline BP	Target BP	Main findings
Vedel et al. (2018) [16]	Randomized controlled trial	197 patients undergoing cardiac surgery under CPB	/	/	High pressure group: MAP 70–80 mmHg Low pressure group: MAP 40–50 mmHg during CPB	Targeting a higher versus lower MAP during CPB did not seem to affect the volume or number of new cerebral infarcts.
Monk et al. (2015) [28]	Retrospective cohort study	18,576 patients undergoing noncardiac surgery	Systolic BP < 90 mmHg, MAP < 60 mmHg, diastolic BP < 50 mmHg, or ↓>30, 40, 50% from the baseline, respectively	The average of all noninvasive BP measurements before the appearance of end-tidal carbon dioxide	/	IOH, defined as systolic BP < 70 mmHg, MAP < 50 mmHg, diastolic BP < 30 mmHg, MAP ↓ >50% from the baseline for ≥5 min, is associated with high operative morbidity and 30-day mortality.
Salmasi et al. (2017) [52]	Retrospective cohort study	53,315 patients undergoing noncardiac surgery	MAP < 75, 70, 65, 60, 55 mmHg MAP ↓ >10, 15, 20, 25% from the baseline	The average of all MAP readings in the 6 months before surgery	/	MAP < 65 mmHg for more than 13 min or a cumulative time exceeding 90 min with a MAP less than 20% below the baseline was related to MINS and AKI. Both absolute and relative MAP thresholds had comparable ability to discriminate patients with MINS or AKI.
Hallqvist et al. (2018) [53]	Observational study	23,140 patients undergoing major noncardiac surgery	Systolic BP ↓ >40 or 50% from the baseline, and lasting more than 5 min	The average of all MAP readings within 2 preoperative months	/	Reduction of systolic BP more than 40% from the baseline was associated with an elevated risk of AKI. Reduction of more than 50% was associated with a more than doubled risk of AKI.
Sessler et al. (2018) [54]	Retrospective cohort study	9765 patients undergoing noncardiac surgery	Systolic BP < 90 mmHg requiring treatment	/	/	IOH and POH were significantly and independently associated with the composite outcomes of myocardial infarction and death within 30 days.
Walsh et al. (2013) [55]	Observational study	33,330 patients undergoing noncardiac surgery	MAP < 55–75 mmHg	/	/	MAP < 55 mmHg even for short durations was associated with AKI and MINS. The risk increased with an increasing hypotension duration.
Loffel et al. (2020) [56]	Retrospective cohort analysis	416 patients undergoing noncardiac surgery	MAP < 65 mmHg	/	/	MAP < 65 mmHg, especially 60 mmHg, is associated with an increased risk of AKI.
Sun et al. (2015) [57]	Retrospective cohort study	5127 patients undergoing noncardiac surgery	MAP < 65, 60, 55 mmHg	/	/	AKI was associated with MAP < 60 mmHg for 11–20 min and MAP < 55 mmHg for >10 min.
Joosten et al. (2021) [58]	Historical cohort study	242 patients undergoing liver transplantation	MAP < 65 mmHg	/	/	IOH was independently associated with AKI after liver transplant surgery. The longer the MAP stays below 65 mmHg, the higher the risk of AKI, and the greater the severity.
Ahuja et al. (2020) [59]	Retrospective cohort study	23,140 patients undergoing noncardiac surgery	/	/	/	Systolic BP < 90 mmHg, MAP < 65 mmHg, and PP > 35 mmHg were all related to postoperative AKI, and MAP < 65 mmHg was the most sensitive predictor of postoperative MINS and AKI.
Jang et al. (2019) [60]	Retrospective study	248 patients undergoing femoral neck fracture surgery	Systolic BP < 80 mmHg or MAP < 55–60 mmHg, persisting for more than 5 min	/	/	IOH was an independent risk factor for AKI (OR = 5.14).
Hallqvist et al. (2016) [61]	Observational cohort study	300 patients undergoing major noncardiac surgery	A 50% decrease in systolic BP relative to the baseline and lasting more than 5 min	The average of all MAP readings for the 2 months before surgery	/	An intraoperative reduction in systolic BP of more than 50% from baseline lasting more than 5 min was independently associated with both myocardial damages on postoperative day 1 and MI within 30 days after surgery.
Hallqvist et al. (2021) [62]	Nested case-control study	652 patients undergoing noncardiac surgery	Systolic BP ↓ ≤20, 21–40, 41–50, or > 50 mmHg from baseline	5 on average, documented within 2 months before surgery, obtained from the surgical ward, preoperative anesthetic consultation, or documen4tations from the primary health care	/	IOH as an independent risk factor of perioperative MI. A reduction of 41–50 mmHg from baseline systolic BP was associated with more than a tripled MI risk.
Abbott et al. (2018) [63]	Prospective cohort study	15,109 patients undergoing noncardiac surgery	Systolic BP < 100 mmHg	/	/	Prolonged HR > 100 bpm in combination with SBP < 100 mmHg was associated with an increased risk of MINS. A combination of the lowest HR >55 bpm and highest systolic BP >160 mmHg was also associated with MINS.
van Waes et al. (2016) [64]	Retrospective cohort study	890 patients undergoing vascular surgery	MAP < 50, <60 mmHg, MAP ↓ >30%, 40% from the baseline	Preinduction MAP	/	A 40% decrease from the baseline with a cumulative duration of >30 min was associated with postoperative MINS. Postoperative MI and death within 30 days occurred more often when the MAP was <60 mmHg.
Sang et al. (2020) [65]	Retrospective study	2517 patients with prior coronary stents undergoing noncardiac surgery	MAP ↓ ≥50%, 40%, or 30% rom the baseline or MAP < 70, <60, or < 50 mmHg	Preinduction MAP	/	The predefined levels of IOH were not significantly associated with postoperative MINS, but intraoperative continuous inotrope/vasopressor use was significantly higher in patients with MINS.
Hu et al. (2021) [66]	A prospective randomized controlled trial	322 patients undergoing noncardiac surgery	/	/	/	High MAP (90–100 mmHg) was associated with a shorter delirium span and a higher intraoperative urine volume than low MAP (60–70 mmHg).
Mathis et al. (2020) [67]	Retrospective cohort study	138,021 patients undergoing major noncardiac surgery	MAP < 50 mmHg, 50–54 mmHg, 55–59 mmHg, and 60–64 mmHg or MAP ↓ >40%, 30–40%, and 20–30% from the baseline	Preinduction MAP, measured in the preoperative holding room on the date of surgery	/	There were no associations between IOH and AKI in patients with a low risk. Patients with a medium risk demonstrated associations between severe IOH (MAP < 50 mmHg) and AKI. Patients with the highest risk and mild IOH (MAP <55–59 mmHg) were associated with AKI.
Stapelfeldt et al. (2017) [68]	Retrospective study	152,445 patients undergoing noncardiac surgery	/	/	/	The greater the hypotension duration, the greater the 30-day mortality risk. These exposure time limit sets were shorter in patients with chronic hypertension.
Wu et al. (2017) [69]	Randomized clinical trial	678 patients with chronic hypertension undergoing major gastrointestinal surgery	/	The average of all cuff pressure 2 to 3 days (at least 3 times) before surgery in the ward	Target MAP: Low (65–79 mmHg) Intermediate (80–95 mmHg) High (96–110 mmHg)	Maintaining intraoperative MAP levels to 80–95 mmHg could reduce postoperative AKI after major abdominal surgery.
Gold et al. (1995) [70]	Randomized clinical trial	248 patients undergoing coronary bypass	/	/	High pressure: MAP 80–100 mmHg Low pressure: MAP 50–60 mmHg during CPB	Maintaining a high MAP during CPB could reduce the total mortality rate and the overall incidence of combined cardiac and neurologic complications at 6 months after operation.
Siepe et al. (2011) [71]	Randomized controlled trial	92 patients undergoing coronary bypass	/	/	High pressure: MAP 80–90 mmHg Low pressure: MAP 60–70 mmHg during CPB	Maintaining perfusion pressure at physiologic levels during CPB was associated with less early postoperative cognitive dysfunction and delirium.
Azau et al. (2014) [72]	Randomized controlled trial	300 patients undergoing cardiac surgery under CPB	/	/	High pressure: MAP 75–85 mmHg Control: MAP 50–60 mmHg during CPB	Maintaining a high level of MAP during CPB did not reduce the risk of postoperative AKI or the mortality rate.
Futier et al. (2017) [73]	Randomized clinical trial	298 patients undergoing major noncardiac surgery	/	BP measured at rest in supine position one day before surgery or obtained from the patients' medical records	Individualized treatment: systolic BP within 10% of the baseline BP Standard treatment: systolic BP > 80 mmHg or > 40% baseline	Individualized BP management reduced the incidence of systemic inflammatory response syndrome and renal, cardiovascular, coagulation, and neurological impairment of at least one vital organ system better than routine management.
de la Hoz et al. (2022) [74]	Retrospective cohort study	4984 patients undergoing cardiac surgery	MAP < 65 mmHg	/	Fraction of overall hypotension >80%, 80–60%, <60%	The total duration of IOH (MAP < 65 mmHg) per 10 min exposure was associated with stroke, AKI, or death in patients undergoing cardiac surgery with CPB.
Murabito et al. (2017) [75]	Randomized controlled trial	40 patients undergoing major general surgery	MAP < 65 mmHg	/	MAP < 65 mmHg and hypotension prediction index 50–85	The combined use of the early warning system and hemodynamic algorithm for intraoperative BP management can reduce the incidence of IOH and organ injury.

IOH: intraoperative hypotension; OR: odds ratio; MINS: myocardial injury after noncardiac surgery; AKI: acute kidney injury; MI: myocardial infarction; HR: heart rate; BP: blood pressure; CPB: coronary pulmonary bypass.

## References

[1] Weiser T. G., Haynes A. B., Molina G. (2016). Size and distribution of the global volume of surgery in 2012. *Bulletin of the World Health Organization*.

[2] Weiser T. G., Haynes A. B., Molina G. (2015). Estimate of the global volume of surgery in 2012: an assessment supporting improved health outcomes. *Lancet*.

[3] Williams B., Mancia G., Spiering W. (2018). 2018 ESC/ESH Guidelines for the management of arterial hypertension. *European Heart Journal*.

[4] Brook R. D., Rajagopalan S. (2018). 2017 ACC/AHA/AAPA/ABC/ACPM/AGS/APhA/ASH/ASPC/NMA/PCNA Guideline for the prevention, detection, evaluation, and management of high blood pressure in adults. A report of the American College of Cardiology/American Heart Association Task Force on clinical practice guidelines. *Journal of the American Society of Hypertension*.

[5] Ackland G. L., Brudney C. S., Cecconi M. (2019). Perioperative Quality Initiative consensus statement on the physiology of arterial blood pressure control in perioperative medicine. *British Journal of Anaesthesia*.

[6] Sessler D. I., Bloomstone J. A., Aronson S. (2019). Perioperative Quality Initiative consensus statement on intraoperative blood pressure, risk and outcomes for elective surgery. *British Journal of Anaesthesia*.

[7] Venkatesan S., Myles P. R., Manning H. J. (2017). Cohort study of preoperative blood pressure and risk of 30-day mortality after elective non-cardiac surgery. *British Journal of Anaesthesia*.

[8] Gu W. J., Hou B. L., Kwong J. S. W. (2018). Association between intraoperative hypotension and 30-day mortality, major adverse cardiac events, and acute kidney injury after non-cardiac surgery: a meta-analysis of cohort studies. *International Journal of Cardiology*.

[9] Saugel B., Reese P. C., Sessler D. I. (2019). Automated ambulatory blood pressure measurements and intraoperative hypotension in patients having noncardiac surgery with general anesthesia: a prospective observational study. *Anesthesiology*.

[10] Buijs F. N., León-Mercado L., Guzmán-Ruiz M., Guerrero-Vargas N. N., Romo-Nava F., Buijs R. M. (2016). The circadian system: a regulatory feedback network of periphery and brain. *Physiology (Bethesda, Md.)*.

[11] Johnson P. C. (1986). Autoregulation of blood flow. *Circulation Research*.

[12] Meng L., Wang Y., Zhang L., McDonagh D. L. (2019). Heterogeneity and variability in pressure autoregulation of organ blood flow: lessons learned over 100+ years. *Critical Care Medicine*.

[13] Larsen F. S., Olsen K. S., Hansen B. A., Paulson O. B., Knudsen G. M. (1994). Transcranial Doppler is valid for determination of the lower limit of cerebral blood flow autoregulation. *Stroke*.

[14] Meng L., Hou W., Chui J., Han R., Gelb A. W. (2015). Cardiac output and cerebral blood Flow. *Anesthesiology*.

[15] Ogoh S., Brothers R. M., Barnes Q. (2005). The effect of changes in cardiac output on middle cerebral artery mean blood velocity at rest and during exercise. *Journal of Physiology*.

[16] Vedel A. G., Holmgaard F., Rasmussen L. S. (2018). High-target versus low-target blood pressure management during cardiopulmonary bypass to prevent cerebral injury in cardiac surgery patients: a randomized controlled trial. *Circulation*.

[17] Agham N. D., Chaskar U. M. (2021). Learning and non-learning algorithms for cuffless blood pressure measurement: a review. *Medical and Biological Engineering and Computing*.

[18] Mukkamala R., Stergiou G. S., Avolio A. P. (2022). Cuffless blood pressure measurement. *Annual Review of Biomedical Engineering*.

[19] Bartels K., Esper S. A., Thiele R. H. (2016). Blood pressure monitoring for the Anesthesiologist. *Anesthesia and Analgesia*.

[20] Kaufmann T., Cox E. G. M., Wiersema R. (2020). Non-invasive oscillometric versus invasive arterial blood pressure measurements in critically ill patients: a post hoc analysis of a prospective observational study. *Journal of Critical Care*.

[21] Wax D. B., Lin H. M., Leibowitz A. B. (2011). Invasive and concomitant noninvasive intraoperative blood pressure monitoring: observed differences in measurements and associated therapeutic interventions. *Anesthesiology*.

[22] Avolio A. P., Van Bortel L. M., Boutouyrie P. (2009). Role of pulse pressure amplification in arterial Hypertension. *Hypertension*.

[23] Pauca A. L., Wallenhaupt S. L., Kon N. D., Tucker W. Y. (1992). Does radial artery pressure accurately reflect aortic pressure?. *Chest*.

[24] Kim W. Y., Jun J. H., Huh J. W., Hong S. B., Lim C. M., Koh Y. (2013). Radial to femoral arterial blood pressure differences in septic shock patients receiving high-dose norepinephrine therapy. *Shock*.

[25] Lee M., Weinberg L., Pearce B. (2015). Agreement between radial and femoral arterial blood pressure measurements during orthotopic liver transplantation. *Critical Care and Resuscitation*.

[26] Fuda G., Denault A., Deschamps A. (2016). Risk factors involved in central-to-radial arterial pressure gradient during cardiac surgery. *Anesthesia and Analgesia*.

[27] van Egmond J., Hasenbos M., Crul J. F. (1985). Invasive v. non-invasive measurement of arterial pressure. Comparison of two automatic methods and simultaneously measured direct intra-arterial pressure. *British Journal of Anaesthesia*.

[28] Monk T. G., Bronsert M. R., Henderson W. G., Mangione M. P., Hammermeister K. E. (2015). Association between intraoperative hypotension and hypertension and 30-day postoperative mortality in noncardiac surgery. *Anesthesiology*.

[29] Cheung C. C., Martyn A., Campbell N., Frost S., Khan N. A. (2015). Predictors of intraoperative hypotension and bradycardia. *American Journal of Medicine*.

[30] Bijker J. B., Persoon S., Peelen L. M. (2012). Intraoperative hypotension and perioperative ischemic stroke after general surgery: a nested case-control study. *Anesthesiology*.

[31] Toyama S., Kakumoto M., Morioka M. (2013). Perfusion index derived from a pulse oximeter can predict the incidence of hypotension during spinal anaesthesia for caesarean delivery. *British Journal of Anaesthesia*.

[32] Ard J. L., Kendale S. (2016). Searching for baseline blood pressure: a comparison of blood pressure at three different care points. *Journal of Clinical Neuroscience*.

[33] Hu R., Kalam Y., Broad J., Ho T., Bellomo R. (2020). Decreased mean perfusion pressure as an independent predictor of acute kidney injury after cardiac surgery. *Heart and Vessels*.

[34] Drummond J. C., Blake J. L., Patel P. M., Clopton P., Schulteis G. (2013). An observational study of the influence of "white-coat hypertension" on day-of-surgery blood pressure determinations. *Journal of Neurosurgical Anesthesiology*.

[35] Czernichow S., Zanchetti A., Turnbull F. (2011). The effects of blood pressure reduction and of different blood pressure-lowering regimens on major cardiovascular events according to baseline blood pressure: meta-analysis of randomized trials. *Journal of Hypertension*.

[36] Nuyujukian D. S., Newell M. S., Zhou J. J., Koska J., Reaven P. D. (2022). Baseline blood pressure modifies the role of blood pressure variability in mortality: results from the ACCORD trial. *Diabetes, Obesity & Metabolism*.

[37] Howell S. J., Sear J. W., Foëx P. (2004). Hypertension, hypertensive heart disease and perioperative cardiac risk. *British Journal of Anaesthesia*.

[38] Varon J., Marik P. E. (2000). The diagnosis and management of hypertensive crises. *Chest*.

[39] Rosenman D. J., McDonald F. S., Ebbert J. O., Erwin P. J., LaBella M., Montori V. M. (2008). Clinical consequences of withholding versus administering renin-angiotensin-aldosterone system antagonists in the preoperative period. *Journal of Hospital Medicine*.

[40] Roshanov P. S., Rochwerg B., Patel A. (2017). WithholdingversusContinuing angiotensin-converting enzyme inhibitors or angiotensin ii receptor blockers before noncardiac surgery. *Anesthesiology*.

[41] Vazquez-Narvaez K. G., Ulibarri-Vidales M. (2019). The patient with hypertension and new guidelines for therapy. *Current Opinion in Anaesthesiology*.

[42] Sanders R. D., Hughes F., Shaw A. (2019). Perioperative Quality Initiative consensus statement on preoperative blood pressure, risk and outcomes for elective surgery. *British Journal of Anaesthesia*.

[43] Andersson C., Shilane D., Go A. S. (2014). Beta-Blocker Therapy and Cardiac Events Among Patients With Newly Diagnosed Coronary Heart Disease. *Journal of the American College of Cardiology*.

[44] Fleisher L. A., Fleischmann K. E., Auerbach A. D. (2014). 2014 ACC/AHA guideline on perioperative cardiovascular evaluation and management of patients undergoing noncardiac surgery: a report of the American College of Cardiology/American Heart Association Task Force on practice guidelines. *Journal of the American College of Cardiology*.

[45] Devereaux P. J., Yang H., Yusuf S. (2008). Effects of extended-release metoprolol succinate in patients undergoing non- cardiac surgery (POISE trial): a randomised controlled trial. *Lancet*.

[46] Venkatesan S., Jorgensen M. E., Manning H. J. (2019). Preoperative chronic beta-blocker prescription in elderly patients as a risk factor for postoperative mortality stratified by preoperative blood pressure: a cohort study. *British Journal of Anaesthesia*.

[47] Kertai M. D., Cooter M., Pollard R. J. (2018). Is Compliance With Surgical Care Improvement Project Cardiac (SCIP-Card-2) measures for perioperative *β*-blockers associated with reduced incidence of mortality and cardiovascular-related critical quality indicators after noncardiac surgery?. *Anesthesia and Analgesia*.

[48] Foëx P., Sear J. W. (2018). Perioperative beta-blockade: a conundrum still in need of study!. *Anesthesia and Analgesia*.

[49] Bijker J. B., van Klei W. A., Kappen T. H., van Wolfswinkel L., Moons K. G., Kalkman C. J. (2007). Incidence of intraoperative hypotension as a function of the chosen definition: literature definitions applied to a retrospective cohort using automated data collection. *Anesthesiology*.

[50] van Zuylen M. L., Gribnau A., Admiraal M. (2021). The role of intraoperative hypotension on the development of postoperative cognitive dysfunction: a systematic review. *Journal of Clinical Anesthesia*.

[51] Weinberg L., Li S. Y., Louis M. (2022). Reported definitions of intraoperative hypotension in adults undergoing non-cardiac surgery under general anaesthesia: a review. *BMC Anesthesiology*.

[52] Salmasi V., Maheshwari K., Yang D. (2017). Relationship between intraoperative hypotension, defined by either reduction from baseline or absolute thresholds, and acute kidney and myocardial injury after noncardiac surgery: a retrospective cohort analysis. *Anesthesiology*.

[53] Hallqvist L., Granath F., Huldt E., Bell M. (2018). Intraoperative hypotension is associated with acute kidney injury in noncardiac surgery. *European Journal of Anaesthesiology*.

[54] Sessler D. I., Meyhoff C. S., Zimmerman N. M. (2018). Period-dependent associations between hypotension during and for four days after noncardiac surgery and a composite of myocardial infarction and death: a substudy of the POISE-2 trial. *Anesthesiology*.

[55] Walsh M., Devereaux P. J., Garg A. X., Kurz A., Sessler D. I. (2013). Relationship between intraoperative mean arterial pressure and clinical outcomes after noncardiac surgery: toward an empirical definition of hypotension. *Anesthesiology*.

[56] Loffel L. M., Bachmann K. F., Furrer M. A., Wuethrich P. Y. (2020). Impact of intraoperative hypotension on early postoperative acute kidney injury in cystectomy patients - a retrospective cohort analysis. *Journal of Clinical Anesthesia*.

[57] Sun L. Y., Wijeysundera D. N., Tait G. A., Beattie W. S. (2015). Association of intraoperative hypotension with acute kidney injury after elective noncardiac surgery. *Anesthesiology*.

[58] Joosten A., Lucidi V., Ickx B. (2021). Intraoperative hypotension during liver transplant surgery is associated with postoperative acute kidney injury: a historical cohort study. *BMC Anesthesiology*.

[59] Ahuja S., Mascha E. J., Yang D. (2020). Associations of intraoperative radial arterial systolic, diastolic, mean, and pulse pressures with myocardial and acute kidney injury after noncardiac surgery: a retrospective cohort analysis. *Anesthesiology*.

[60] Jang W. Y., Jung J. K., Lee D. K., Han S. B. (2019). Intraoperative hypotension is a risk factor for postoperative acute kidney injury after femoral neck fracture surgery: a retrospective study. *BMC Musculoskeletal Disorders*.

[61] Hallqvist L., Mårtensson J., Granath F., Sahlén A., Bell M. (2016). Intraoperative hypotension is associated with myocardial damage in noncardiac surgery: an observational study. *European Journal of Anaesthesiology*.

[62] Hallqvist L., Granath F., Fored M., Bell M. (2021). Intraoperative hypotension and myocardial infarction development among high-risk patients undergoing noncardiac surgery: a nested case-control study. *Anesthesia and Analgesia*.

[63] Abbott T. E. F., Pearse R. M., Archbold R. A. (2018). A prospective international multicentre cohort study of intraoperative heart rate and systolic blood pressure and myocardial injury after noncardiac surgery: results of the VISION study. *Anesthesia and Analgesia*.

[64] van Waes J. A., van Klei W. A., Wijeysundera D. N., van Wolfswinkel L., Lindsay T. F., Beattie W. S. (2016). Association between intraoperative hypotension and myocardial injury after vascular surgery. *Anesthesiology*.

[65] Sang H. L., Jie A. K., Heo B. Y., Kim Y. R., Ahn S. (2020). Association between intraoperative hypotension and postoperative myocardial injury in patients with prior coronary stents undergoing high-risk surgery: a retrospective study. *Journal of Anesthesia*.

[66] Hu A. M., Qiu Y., Zhang P. (2021). Higher versus lower mean arterial pressure target management in older patients having non-cardiothoracic surgery: a prospective randomized controlled trial. *Journal of Clinical Anesthesia*.

[67] Mathis M. R., Naik B. I., Freundlich R. E. (2020). Preoperative risk and the association between hypotension and postoperative acute kidney injury. *Anesthesiology*.

[68] Stapelfeldt W. H., Yuan H., Dryden J. K. (2017). The SLUScore: a novel method for detecting hazardous hypotension in adult patients undergoing noncardiac surgical procedures. *Anesthesia and Analgesia*.

[69] Wu X., Jiang Z., Ying J., Han Y., Chen Z. (2017). Optimal blood pressure decreases acute kidney injury after gastrointestinal surgery in elderly hypertensive patients: a randomized study: optimal blood pressure reduces acute kidney injury. *Journal of Clinical Anesthesia*.

[70] Gold J. P., Charlson M. E., Williams-Russo P. (1995). Improvement of outcomes after coronary artery bypass: A randomized trial comparing intraoperative high versus low mean arterial pressure. *Journal of Thoracic and Cardiovascular Surgery*.

[71] Siepe M., Pfeiffer T., Gieringer A. (2011). Increased systemic perfusion pressure during cardiopulmonary bypass is associated with less early postoperative cognitive dysfunction and delirium. *European Journal of Cardio-Thoracic Surgery*.

[72] Azau A., Markowicz P., Corbeau J. J. (2014). Increasing mean arterial pressure during cardiac surgery does not reduce the rate of postoperative acute kidney injury. *Perfusion*.

[73] Futier E., Lefrant J. Y., Guinot P. G. (2017). Effect of individualized vs standard blood pressure management strategies on postoperative organ dysfunction among high-risk patients undergoing major surgery: a randomized clinical trial. *JAMA*.

[74] de la Hoz M. A., Rangasamy V., Bastos A. B. (2022). Intraoperative hypotension and acute kidney injury, stroke, and mortality during and outside cardiopulmonary bypass: a retrospective observational cohort study. *Anesthesiology*.

[75] Murabito P., Astuto M., Sanfilippo F. (2022). Proactive management of intraoperative hypotension reduces biomarkers of organ injury and oxidative stress during elective non-cardiac surgery: a pilot randomized controlled trial. *Journal of Clinical Medicine*.

[76] Gregory A., Stapelfeldt W. H., Khanna A. K. (2021). Intraoperative hypotension is associated with adverse clinical outcomes after noncardiac surgery. *Anesthesia and Analgesia*.

[77] Wesselink E. M., Kappen T. H., Torn H. M., Slooter A. J. C., van Klei W. A. (2018). Intraoperative hypotension and the risk of postoperative adverse outcomes: a systematic review. *British Journal of Anaesthesia*.

[78] Palmer B. F. (2002). Renal dysfunction complicating the treatment of hypertension. *New England Journal of Medicine*.

[79] Polese A., De Cesare N., Montorsi P. (1991). Upward shift of the lower range of coronary flow autoregulation in hypertensive patients with hypertrophy of the left ventricle. *Circulation*.

[80] Almeida J. B., Saragoça M. A., Tavares A., Cezareti M. L., Draibe S. A., Ramos O. L. (1992). Severe hypertension induces disturbances of renal autoregulation. *Hypertension*.

[81] Briesenick L., Flick M., Saugel B. (2021). Postoperative blood pressure management in patients treated in the ICU after noncardiac surgery. *Current Opinion in Critical Care*.

[82] Liem V. G. B., Hoeks S. E., Mol K. (2020). Postoperative hypotension after noncardiac surgery and the association with myocardial injury. *Anesthesiology*.

[83] van Lier F., Wesdorp F. H. I. M., Liem V. G. B. (2018). Association between postoperative mean arterial blood pressure and myocardial injury after noncardiac surgery. *British Journal of Anaesthesia*.

[84] McEvoy M. D., Gupta R., Koepke E. J. (2019). Perioperative Quality Initiative consensus statement on postoperative blood pressure, risk and outcomes for elective surgery. *British Journal of Anaesthesia*.

[85] Mohammed Iddrisu S., Considine J., Hutchinson A. (2018). Frequency, nature and timing of clinical deterioration in the early postoperative period. *Journal of Clinical Nursing*.

[86] Kause J., Smith G., Prytherch D., Parr M., Flabouris A., Hillman K. (2004). A comparison of antecedents to cardiac arrests, deaths and emergency intensive care admissions in Australia and New Zealand, and the United Kingdom--the ACADEMIA study. *Resuscitation*.

[87] Liu Y. L., John P., Elisa L., Shigehiko U., Rinaldo B. (2008). Changes in blood pressure before the development of nosocomial acute kidney injury. *Nephrology, Dialysis, Transplantation*.

[88] Smischney N. J., Shaw A. D., Stapelfeldt W. H. (2020). Postoperative hypotension in patients discharged to the intensive care unit after non-cardiac surgery is associated with adverse clinical outcomes. *Critical Care*.

[89] Khanna A. K., Maheshwari K., Mao G. (2019). Association between mean arterial pressure and acute kidney injury and a composite of myocardial injury and mortality in postoperative critically ill patients: a retrospective cohort analysis. *Critical Care Medicine*.

[90] Khanna A. K., Shaw A. D., Stapelfeldt W. H. (2021). Postoperative hypotension and adverse clinical outcomes in patients without intraoperative hypotension, after noncardiac surgery. *Anesthesia and Analgesia*.

[91] Turan A., Chang C., Cohen B. (2019). Incidence, severity, and detection of blood pressure perturbations after abdominal surgery: a prospective blinded observational study. *Anesthesiology*.

[92] Mcgillion M. H., Duceppe E., Allan K., Marcucci M., Devereaux P. J. (2018). Postoperative remote automated monitoring: need for and state of the science. *Canadian Journal of Cardiology*.

[93] Michard F., Bellomo R., Taenzer A. (2019). The rise of ward monitoring: opportunities and challenges for critical care specialists. *Intensive Care Medicine*.

[94] Khanna A. K., Hoppe P., Saugel B. (2019). Automated continuous noninvasive ward monitoring: future directions and challenges. *Critical Care*.

[95] Williamson J. D., Supiano M. A., Applegate W. B. (2016). Intensive vs standard blood pressure control and cardiovascular disease outcomes in adults aged ≥75 years: a randomized clinical trial. *JAMA*.

[96] Croall I. D., Tozer D. J., Moynihan B. (2018). Effect of standard vs intensive blood pressure control on cerebral blood flow in small vessel disease: the PRESERVE randomized clinical trial. *JAMA Neurology*.

[97] Nicklas J. Y., Diener O., Leistenschneider M. (2020). Personalised haemodynamic management targeting baseline cardiac index in high- risk patients undergoing major abdominal surgery: a randomised single-centre clinical trial. *British Journal of Anaesthesia*.

[98] Godet T., Grobost R., Futier E. (2018). Personalization of arterial pressure in the perioperative period. *Current Opinion in Critical Care*.

[99] Nasrallah I. M., Gaussoin S. A., Pomponio R. (2021). Association of intensive vs standard blood pressure control with magnetic resonance imaging biomarkers of alzheimer disease: secondary analysis of the SPRINT MIND randomized trial. *JAMA Neurology*.

[100] Gottesman O., Scott S. A., Ellis S. B. (2013). The CLIPMERGE PGx program: clinical implementation of personalized medicine through electronic health records and genomics-pharmacogenomics. *Clinical Pharmacology and Therapeutics*.

[101] Joosten A., Rinehart J., Van der Linden P. (2021). Computer-assisted individualized hemodynamic management reduces intraoperative hypotension in intermediate- and high-risk surgery: a randomized controlled trial. *Anesthesiology*.

[102] Hatib F., Jian Z., Buddi S. (2018). Machine-learning algorithm to predict hypotension based on high-fidelity arterial pressure waveform analysis. *Anesthesiology*.

[103] Schneck E., Schulte D., Habig L. (2020). Hypotension Prediction Index based protocolized haemodynamic management reduces the incidence and duration of intraoperative hypotension in primary total hip arthroplasty: a single centre feasibility randomised blinded prospective interventional trial. *Journal of Clinical Monitoring and Computing*.

[104] Maheshwari K., Shimada T., Yang D. (2020). Hypotension prediction index for prevention of hypotension during moderate- to high-risk noncardiac surgery. *Anesthesiology*.

[105] Joosten A., Vincent J. L., Saugel B. (2020). Continuous non-invasive haemodynamic monitoring in patients having surgery: valuable tool or superfluous toy?. *Anaesthesia, Critical Care & Pain Medicine*.

[106] Alexander B., Rinehart J., Cannesson M., Duranteau J., Joosten A. (2019). Closed-loop hemodynamic management. *Best Practice & Research. Clinical Anaesthesiology*.

[107] Rinehart J., Lee S., Saugel B., Joosten A. (2021). Automated blood pressure control. *Seminars in Respiratory and Critical Care Medicine*.

[108] Saugel B., Kouz K., Scheeren T. W. L. (2019). The ‘5 Ts’ of perioperative goal-directed haemodynamic therapy. *British Journal of Anaesthesia*.

[109] Fellahi J. L., Futier E., Vaisse C. (2021). Perioperative hemodynamic optimization: from guidelines to implementation-an experts' opinion paper. *Annals of Intensive Care*.

[110] Wu X., Jiang Z., Chen Z. (2018). Intraoperative mean arterial pressure: what is the magic level really favorable for renal function?. *Journal of Clinical Anesthesia*.

[111] London M. J. (2016). Intraoperative mean blood pressure and Outcome. *Anesthesiology*.

[112] Wijnberge M., Schenk J., Bulle E. (2021). Association of intraoperative hypotension with postoperative morbidity and mortality: systematic review and meta-analysis. *BJS Open*.

[113] Vernooij L. M., van Klei W. A., Machina M., Pasma W., Beattie W. S., Peelen L. M. (2018). Different methods of modelling intraoperative hypotension and their association with postoperative complications in patients undergoing non-cardiac surgery. *British Journal of Anaesthesia*.

[114] Holte K., Foss N. B., Svensén C., Lund C., Madsen J. L., Kehlet H. (2004). Epidural anesthesia, hypotension, and changes in intravascular volume. *Anesthesiology*.

[115] Vincent J. L. (2020). Intravascular volume assessment in the critically ill patient. *Clinical Journal of the American Society of Nephrology*.

[116] Tu M. Y., Hong S., Lu J., Liu Y. H., Deng M. (2021). Effect of strict intraoperative blood pressure management strategy on postoperative acute kidney injury in non-cardiac surgery: a meta-analysis of randomised controlled trials. *International Journal of Clinical Practice*.

[117] Brown C. H., Neufeld K. J., Tian J. (2019). Effect of targeting mean arterial pressure during cardiopulmonary bypass by monitoring cerebral autoregulation on postsurgical delirium among older patients: a nested randomized clinical trial. *JAMA Surgery*.

[118] Charlson M. E., MacKenzie C. R., Gold J. P., Ales K. L., Topkins M., Shires G. T. (1990). Intraoperative blood pressure. What patterns identify patients at risk for postoperative complications?. *Annals of Surgery*.

[119] Fumagalli U., Melis A., Balazova J., Lascari V., Morenghi E., Rosati R. (2016). Intra-operative hypotensive episodes may be associated with post-operative esophageal anastomotic leak. *Updates in Surgery*.

[120] Reich D. L., Bennett-Guerrero E., Bodian C. A., Hossain S., Winfree W., Krol M. (2002). Intraoperative tachycardia and hypertension are independently associated with adverse outcome in noncardiac surgery of long duration. *Anesthesia and Analgesia*.

[121] Aronson S., Stafford-Smith M., Phillips-Bute B. (2010). Intraoperative systolic blood pressure variability predicts 30-day mortality in aortocoronary bypass surgery patients. *Anesthesiology*.

[122] Ono M., Brady K., Easley R. B. (2014). Duration and magnitude of blood pressure below cerebral autoregulation threshold during cardiopulmonary bypass is associated with major morbidity and operative mortality. *Journal of Thoracic and Cardiovascular Surgery*.

[123] McEwen C. C., Amir T., Qiu Y. (2022). Morbidity and mortality in patients managed with high compared with low blood pressure targets during on-pump cardiac surgery: a systematic review and meta-analysis of randomized controlled trials. *Canadian Journal of Anaesthesia*.

